RETRACTED

# Fatal Prion Disease in a Mouse Model of Genetic E200K Creutzfeldt-Jakob Disease

**DOI:** 10.1371/journal.ppat.1002350

**Published:** 2011-11-03

**Authors:** Yael Friedman-Levi, Zeev Meiner, Tamar Canello, Kati Frid, Gabor G. Kovacs, Herbert Budka, Dana Avrahami, Ruth Gabizon

**Affiliations:** 1 Department of Neurology, The Agnes Ginges Center for Human Neurogenetics, Jerusalem, Israel; 2 Institute of Neurology, Medical University Vienna, Austria; University of Alberta, Canada

## Abstract

Genetic prion diseases are late onset fatal neurodegenerative disorders linked to pathogenic mutations in the prion protein-encoding gene, *PRNP*. The most prevalent of these is the substitution of Glutamate for Lysine at codon 200 (E200K), causing genetic Creutzfeldt-Jakob disease (gCJD) in several clusters, including Jews of Libyan origin. Investigating the pathogenesis of genetic CJD, as well as developing prophylactic treatments for young asymptomatic carriers of this and other PrP mutations, may well depend upon the availability of appropriate animal models in which long term treatments can be evaluated for efficacy and toxicity. Here we present the first effective mouse model for E200KCJD, which expresses chimeric mouse/human (TgMHu2M) E199KPrP on both a null and a wt PrP background, as is the case for heterozygous patients and carriers. Mice from both lines suffered from distinct neurological symptoms as early as 5–6 month of age and deteriorated to death several months thereafter. Histopathological examination of the brain and spinal cord revealed early gliosis and age-related intraneuronal deposition of disease-associated PrP similarly to human E200K gCJD. Concomitantly we detected aggregated, proteinase K resistant, truncated and oxidized PrP forms on immunoblots. Inoculation of brain extracts from TgMHu2ME199K mice readily induced, the first time for any mutant prion transgenic model, a distinct fatal prion disease in wt mice. We believe that these mice may serve as an ideal platform for the investigation of the pathogenesis of genetic prion disease and thus for the monitoring of anti-prion treatments.

## Author Summary

Inherited prion diseases, such as genetic CJD, are dominant disorders linked to mutations in the gene encoding the prion protein, PrP. Since therapeutic intervention in all types of human prion diseases has failed, we propose that therapeutic efforts should be directed mostly to the development of preventive treatments for subjects incubating prion diseases, as is the case for asymptomatic carriers of pathogenic PrP mutations. These subjects will develop disease symptoms at some point in their adult life; therefore they should be treated before clinical deterioration. Candidate treatments will need to be tested for efficacy and safety first in animal models that mimic most properties of genetic CJD. In this work, we describe a new transgenic mouse model for E200K genetic CJD, presenting progressive neurodegenerative disease and age related prion disease pathology and biochemistry, as is the case in the human disease. Brain extracts from these mice also transmitted prion disease to wt mice, as shown before for parallel human samples. We propose that these animals will play a significant role in the development of novel anti-prion prophylactic treatments.

RETRACTED

## Introduction

Inherited prion diseases, such as gCJD and Gerstmann–Sträussler–Scheinker (GSS), are autosomal dominant disorders linked to mutations in the gene encoding the prion protein (PrP), denominated *PRNP* [1], [2]. The largest focus of gCJD was identified among Libyan Jews carrying a missense mutation in codon 200 of *PRNP* (substituting lysine for glutamate, E200K) [3], [4]. This same mutation was also found in other communities around the world [5].

As of today, therapeutic intervention in human prion diseases has failed [6] [7]. Indeed, some protocols reduced the rate of patients' deterioration for short periods of time [8], but none could hope to reverse the severe neurological deficits apparent already at diagnosis. We therefore propose that efforts should be directed mostly to develop preventive treatments for subjects at risk, as is the case for asymptomatic carriers of genetic prion diseases. Candidate anti-prion reagents will need to be tested in transgenic models mimicking gCJD. Such transgenic mice should succumb spontaneously to neurological disease in a high attack rate and in a short time frame, allowing for long term treatments and measurable delay of onset well within the life span of the animals. The model mice should also present prion related biochemistry and pathology, and if possible transmit disease directly to wt animals, as is the case for humans suffering from gCJD [9] [10].

Indeed, several animal models of genetic prion disease were generated in the past, thereby demonstrating that late onset and spontaneous genetic human prion diseases can be reconstructed in mice [11], [12]. While very useful in the study of prion disease pathogenesis, not all these models presented all the properties described above.

The first transgenic (Tg) mice imitating human genetic prion disease carried a P102L-PrP GSS mutation on a mouse background and succumb spontaneously to prion disease after about 4–6 months [13]. However these mice transmitted infectivity only to unique recipients [14], [15], and in addition presented poor PrP pathology. Tg lines mimicking the PrP insertional mutation [16], the A117V mutation [17], as well as both the CJD [18] and the FFI D178N [19] mutation presented prion-like clinical disease with low to marginal disease related PrP. The FFI D178N mice transmitted disease to mice overexpressing wtPrP as well as those expressing wtPrP with the 3F4 epitope, and the recipient mice developed prion-related neuropathology in the absence of disease related PrP [19]. Two Tg lines mimicking the E200K PrP mutation, one on a human PrP gene and another on a mouse PrP gene did not present disease or other prion related properties [20] [21].

RETRACTED

In this work, we describe a transgenic mouse model for E200K gCJD expressing a chimeric mouse/human PrP [15], [22] both on a wt and a null PrP background, hereby denominated TgMHu_2_ME199K/wt and TgMHu2ME199K/ko respectively. The line on the wt background mimics most gCJD patients, who are heterozygous for the PrP mutation [2]. Mice from both lines presented progressive neurodegenerative disease starting from 5 to 6 month of age, deteriorated and died several months thereafter. Their brains comprise age related pathology characteristic of prion disease, such as gliosis and accumulated disease related PrP, which was shown by immunoblots to be resistant to digestion by high concentrations of proteinase K (PK). Most important, brain extracts from both lines transmitted prion disease to wt mice. We believe that these animals will play a significant role in the investigation of genetic prion disease pathogenesis and most important, in the development of novel anti-prion prophylactic treatments.

## Results

### TgMHu2ME199K mice develop spontaneous progressive neurological disease

TgMHu2ME199K on both a wt and a PrP ablated background were constructed (as described in the methods) by inserting an E to K substitution at position 199 of a chimeric mouse human (MHu_2_M) PrP construct. As of today a total of 300 mice were generated (240 on an ablated background and 60 on a wt background), and used for the different experiments described in this manuscript. These include characterization of clinical disease as well as investigation of kinetic of disease progression. We also studied pathological and biochemical prion disease properties of the Tg mice at different time points before and throughout disease progression and collected samples for expression and transmission studies.

The most prominent symptom of disease, which appeared in all Tg MHu_2_M E199K mice already at 5–6 months of age, is an a-symmetric hind limbs weakness that develops with time to paraplegia. This sign was followed by leg clasping and lower body atrophy. Contrarily, some of the most characteristic clinical signs of prion symptoms, i.e. plastic tail and tremor were only apparent in some of the mice. Figure 1 depicts affected mice suffering from hind limbs plegia, lower body atrophy and leg clasping. While the mice in the figure are each from a different line (Tg/ko and Tg/wt), the different signs appear in all sick mice. The clinical symptoms of the TgMHu2ME199K mice by order of appearance are described in Table 1. Table 2 demonstrates the score we constructed out of these clinical symptoms for kinetic analysis of disease progression. The time point of death (score 5) was determined when a mouse was too paralyzed to reach food and water independently (according to local committee ethical requirements).

RETRACTED

**Figure 1:** Clinical Characterization of spontaneous disease in TgMHu2ME199K mice. Typical pictures of sick TgMHu2ME199K mice showing hind limbs plegia, kyphosis and leg clasping.

**Table 1:** Clinical signs by order of appearance.

	Percentage of affected mice
A-symmetric hind limbs weakness	100%
A-symmetric hind limbs plegia	100%
Abnormal hind limbs posture	100%
Lower body atrophy	100%
Kyphosis	100%
Myoclonic jerks	∼10%
Tremor	∼20%
Plastic tail	Rare (less than 5%)
Blindness	Rare (less than 5%)

**Table 2:** Score of disease severity by clinical signs.

Hind limbs weakness	1
Hind limbs partial paralysis	2
Full paralysis in one limb	3
Full hind limbs paralysis	4
Death	5

Additional symptoms such as plastic tail (rare) or tremor added one point to the total score.

To evaluate the kinetics of disease progression in these mice, a designated group of 62 TgMHu2ME199K/ko and 14 TgMHu2ME199K/wt, (half male, and half female) was followed carefully from birth throughout disease progression to death. Figure 2a shows the average age of disease onset (score 1) and disease end point (score 5) in the transgenic mice. Figure 2 b presents the severity of disease as related to age (each point represent the average score in groups of 2–8 littermates, which were averaged together to avoid individual differences), while figure 2 c demonstrates disease prevalence in these same groups as related to age. As stated above, our results indicate that all TgMHu2ME199K mice demonstrate first disease symptoms between the ages of 5 to 7 months old. No significant differences were observed in clinical and kinetic parameters between male and female mice. Small differences (non significant) in disease presentation and progression were observed between mice expressing the chimeric mutant PrP on null as compared to wt PrP background (figure 2a), however this may result from the smaller numbers of mice in the TgMHu2ME199K/wt group. Additional transgenic mice used in time course experiments showed similar disease parameters.

RETRACTED

**Figure 2:** Disease progression in spontaneous disease. **a:** Average disease onset and death of mice in kinetic studies. **b:** Aggravation of clinical score of disease as related to the mice's age and gender. Groups of TgMHu2ME199K mice (male and female) were scored for clinical signs from birth to death. Average disease score for each group was plotted against the age elapsed since the mice birth. Closed circles: males, open circles: females. **c:** Percentage of sick mice in each age group. Groups of mice (as in fig b) in which the average score was at least 1 were plotted against the age of the mice. Closed circles: males, open circles: females **d:** Relative PrP mRNA levels, as determined by quantitative RT-PCR for wt and TgMHu2ME199K/ko mice. Each bar represents the average of PrP mRNA normalized against controls genes levels (see methods) in 4 male mice. Statistical bars represent standard error **e:** Brain homogenates from TgMHu2ME199K/ko, TgMHu2ME199K/wt, PrP ablated, wt C57BL/6 and RML-infected mice were immunoblotted with α PrP 6H4 mAb **f:** Relative intensities of the bands as measured by NIH Image J analysis software.

### PrP expression in TgMHu2ME199K mice

We next investigated the levels of PrP expression in the brains of the TgMHu2ME199K mice. To this effect, mRNA samples purified from brains of wt and TgMHu2ME199K/ko 6 months old mice (4 for each group) were subjected to reverse transcriptase and subsequently to amplification by real time PCR of PrP and control genes (see methods). Figure 2d shows that while mRNA levels of PrP were 20 fold higher in the brains of the transgenic mice as compared to wt mice, the actual levels of the PrP protein, as tested by immunoblotting of brain homogenates with α PrP mAb 6H4, were only increased by 2 folds (figures 2e &f). Whether this discrepancy between the PrP mRNA and protein levels of mutant PrP in the Tg mice is of biological significance is unknown at this point.

### Neuropathological evaluation of the spontaneous prion disease in TgMHu2ME199K mice

Four µm thick sections of formalin-fixed, paraffin-embedded brains and spinal cords of TgMHu2ME199K mice of different ages and gene array were evaluated for neuropathology and PrP immunoreactivity with different α PrP antibodies (see figure 3a for epitope description of all α PrP antibodies used in this project). Figure 3b depicts the results for 8 months old mice (at least 3 in each group) of the different lines (TgMHu_2_ME199K/ko, TgMHu2ME199K/wt, PrP^0/0^ and wt mice). Figure S1 presents results for TgMHu2ME199K/ko mice at different ages (3 in each group), which are also summarized in figure 4. None of the Tg mice brains exhibited inflammatory infiltrates, demyelination, axonal swellings, or abnormal neurites, in accordance with classical prion disease–related pathology [23].

RETRACTED

**Figure 3:** PrP immunoreactivity in the brains of TgMHu2ME199K mice. **a:** Epitope mapping of α PrP antibodies used in these experiments. **b:** Four µm thick sections of formalin fixed, paraffin embedded brains from 8 months old TgMHu2ME199K on wt and ablated background, as compared to wt and PrP ablated mice were tested for disease related PrP immunoreactivity in diverse brain regions with both α PrP pAb RTC and α PrP mAb 6H4. The figure represents at least 3 samples from each group, and depicts intracellular PrP staining with RTC for the sick Tg mice. Scale bar in the upper left panel indicates 20 µm.

**Figure 4:** Summary of Pathology of TgMHu2ME199K mice: time course. This figure summarizes the pathological findings in TgMHu2ME199K/ko mice of different ages (at least 3 mice for each age group, see Figure S1) **a:** the score for gliosis/neuronal loss in different brain areas of the TgMHu2ME199K mice as a function of aging. **b:** intraneuronal PrP immunoreactivity score in different brain areas as a function of aging.

The predominant form of disease related PrP immunoreactivity in the TgMHu2ME199K mice was an intraneuronal dot-like and granular immunostaining in widespread distribution but mainly in neurons of the spinal cord, basal ganglia, thalamus, frontal cortex, and in brainstem nuclei. This was detected by the C-terminally directed αPrP pAb RTC, and less so by αPrP mAb 12F10 (shown for human in Figure S1). Plaque-like or coarse PrP immunoreactivity was not seen in any of the sick TgMHu2ME199K mice. These patterns of immunopositivity, in particular the intraneuronal staining, is strikingly reminiscent of recently described human E200K gCJD [24]. In addition to the intraneuronal PrP detected by RTC, a fine granular immunostaining reminiscent of the so-called synaptic immunoreactivity was observed by immunostaining for α PrP mAb 6H4 (figure 3b and figure S1). Interestingly, while the intraneuronal PrP immunoreactivity was prominent in many regions including the spinal cord, the synaptic type was rather seen in subcortical gray matter structures (see figure S1 and figure 4 for time course and summary of pathological results). Both forms of disease-associated PrP immunodeposits are present in humans affected by E200K linked gCJD [24], further supporting the similarity between the human disease and this animal model.

For technical reasons, the pathological examination of heterozygous E200K human patients [24] could not establish whether the intracellular staining was associated with E200K PrP, wtPrP or both PrP forms. However, the examination of our TG model, which allows for the comparison of Tg/ko with Tg/wt, provides a partial answer to this question. Since there was no apparent difference between the PrP immunoreactivity of both these lines with RTC and 6H4 (figure 3), we may conclude that mutant PrP thus accumulate intraneuronally in all sick Tg mice. To establish whether also wt PrP in the TgMHu2ME199K/wt mice can accumulate inside neurons or produce any form of disease related PrP, we need an antibody that will recognize only this PrP form. Regretfully, we could not allocate a reagent with exclusive specificity for wt PrP as opposed to MHu2M PrP that will also be suitable for pathological studies.

RETRACTED

Spongiform changes, a common feature of scrapie RML strain in mice [25], were observed only focally at the end-stage of disease, mostly in the frontal cortex and in the basal ganglia (figure S1). Mild degree of neuronal loss and reactive astrogliosis was observed already in 3 months old Tg mice in the basal ganglia, thalamus, and circumscribed areas of the frontal cortex, as well as in the spinal cord. These alterations became more prominent in later stages (at 8 months old and at the end point of disease) concomitantly with the clinical symptoms described above (see figure S1 and figure 4).

### Biochemical characterization of PrP in the spontaneous disease

As described above, intraneuronal PrP in the TgMHu2ME199K mice was visualized mostly with C-terminal αPrP antibodies, in particular RTC, a polyclonal antibody which detects the 201–205 PrP epitope [26], suggesting disease related PrP may accumulate in the Tg mice as an N-terminally truncated form. To further test this possibility by biochemical methods, as well as to evaluate other prion like biochemical properties of PrP in the Tg mice, we used diverse αPrP antibodies (see figure 3a for specific epitopes) to immunoblot brain homogenates from 8 months old mice from different genetic backgrounds (figure 5a). These include TgMHu_2_M E200K mice on both the ablated (lane 1) and wt (lane 2) PrP background, as well as from age matched wt TgMHu_2_M (wt chimeric human *PRNP* transgene mice (lane 3), which have not developed spontaneous neurological disease during their life span [15]. As additional controls, we also tested brain homogenates from normal (lane 4) and RML scrapie infected (lane 5) mice (also see insert in figure 5 for sample description). Panel 5a shows that while αPrP mAb IPC1 reacted preferentially with samples 2, 4, and 5 which express PrP from a wt mouse allele, mAb 3F4 reacted only with the samples expressing TgMHu_2_MPrP, regardless of the presence of the E200K mutation or of the additional expression of wt PrP. Contrarily to the antibodies with species selective immunoreactivity (IPC1 and 3F4), mAb 6H4 recognized PrP forms from all brain samples at comparable levels (see also figure 1c). Last, the C-terminal RTC antibody detected equally the established PrP bands in all samples, but in addition recognized some truncated PrP forms (of about 10 and 20 kDA) in the samples comprising a TgMHu2ME199K allele. These bands (see arrows for truncated forms) were absent from samples of both wt mice and TgMHu_2_M controls, suggesting they are specific for PrP in the TgMHu2ME199K mice.

RETRACTED

**Figure 5:** Biochemical Characterization of PrP in TgMHu2ME199K mice. **a:** To establish the PrP specificity of different samples, brain homogenates from 8 months old mice from 1: TgMHu2ME199K/ko, 2: TgMHu2ME199K/wt, 3: TgMHu_2_M, 4: wt C57BL/6, and 5: RML infected mice, were immunoblotted with several α PrP antibodies (See figure 3a for α PrP epitope mapping). Arrows demonstrate truncated PrP forms only present in brains of TgMHu2ME199K mice. **b:** Samples as in panel a were treated in the presence or absence of PNGase and immunoblotted with designated α PrP antibodies. As above truncated PrP forms are demonstrated only in the TgMHu2ME199K mice demonstrated with arrows. **c:** Samples as in panel a were extracted with sarkosyl and then centrifuged at 100000 g for 1 h, separated into pellets and supernatants. Otherwise, similar samples (denominated as total) were digested with 30 ug/ml PK for 30 min at 37°C. All samples were then immunoblotted with the designated anti PrP antibodies. Arrows demonstrate PK resistant bands in the TgMHu2ME199K samples. **d:** Samples from TgMHu2ME199K/ko mice at different ages and controls were digested in the presence or absence of 30 ug/ml PK for 30 min at 37°C and immunoblotted with α PrP pAb RTC. #1: 1 month old; #2: 3 months old; #3: 7 months old; #4: another 7 months old sample, #5 PrP ablated mouse; #6 wt mouse, #7 RML infected mouse.

To learn more about the PrP bands recognized by pAb RTC in the Tg mice brains, we subjected the samples presented in panel a to digestion by PNGase, an enzyme which removes N-linked sugars from proteins [27]. Figure 5b shows that while the 26 KDa band, representing deglycosylated full length PrP was detected by RTC in all samples, the TgMHu2ME199K samples presented additional and unique deglycosylated bands (see arrows), different also in their molecular weight from the 19 Kda band representing deglycosylated PK resistant PrP in scrapie brains (lane 5).

To investigate whether PrP forms present in the brains of sick TgMHu2ME199K mice are aggregated and PK resistant, properties established as the hallmark of disease related PrP, we subjected Sarkosyl extracted brain homogenates from sick TgMHu2ME199K mice and controls (same lane numbering as above) to centrifugation at 100,000 g. In parallel, similar homogenate samples were digested with 30 µg/ml PK for 30 minutes at 37°C. The samples generated by these experiments were immunoblotted with α PrP antibodies 6H4 and RTC. Figure 5c shows that a significant fraction of the PrP protein present in the sick mice (lanes 1&2) pelleted under these conditions, resembling the fraction of aggregated PrP in scrapie infected mice (lane 5). This was not the case for PrP in the samples from the control chimeric or from the wt mice (lanes 3&4). As in the previous panel, immunoblotting of the same samples with pAb RTC revealed additional lower bands of about 10 to 20 Kda, in both the pellet and the supernatant. Following digestion of the homogenates with PK, and consistent with the pathological results (figure 2); it was again RTC that could detect the PrP bands resistant to protease digestion.

RETRACTED

To establish whether truncated PK resistant PrP in the brains of TgMHu2ME199K mice are a feature of the mutated PrP chimera at all ages or represent the onset of disease in older mice, we looked for their presence in the brains of young and asymptomatic TgMHu2ME199K mice. Figure 5d shows that PK resistant PrP was absent at 1 month of age (lane 1), barely present at 3 months of age (lane 2), but was clearly apparent at 8 months of age (lanes 3 and 4), when animals were severely sick. These results demonstrate that, consistent with the immunohistochemistry results described in figure 4, the appearance of PK resistant PrP forms correlate with age and disease progression, and are not an automatic feature of mutated PrP.

### Oxidation properties of PrP in the spontaneous and the transmitted disease

We have recently shown that pAb RVC, a polyclonal antibody generated against reduced 203–214 human/mouse PrP peptides, could not detect Human PrP^Sc^ in brains of genetic or sporadic CJD patients [26]. This and other experiments demonstrated that Methionine residues (Met) in human PrP^Sc^ are present in an oxidized form. This was also the case for Met residues in recombinant human E200K PrP. To test the oxidation status of PrP in our sick TgMHu2ME199K mice, we subjected Sarkosyl extracted brain homogenates from wt and from TgMHu2ME199K/ko mice, as well as from mice infected with RML prions to 10–60% sucrose gradients. Subsequently, the gradient fractions were immunoblotted with both RTC and RVC α PrP antibodies. Figure 6 shows how PrP in the TgMHu2ME199K mice (both full length and truncated) was detected in all the gradients fractions when the blots were challenged with pAb RTC, indicating the mutant protein may be present in the brains of these mice at diverse aggregation states. In contrast, pAb RVC detected only full length PrP in the lighter fractions, suggesting that TgMHu2ME199K PrP may be oxidized and aggregated during its metabolic pathway in the Tg mice, as is also the case for PrP^Sc^ in the infected brains. These experiments indicate that most mutant PrP in the Tg mice is not oxidized immediately upon its generation, but becomes oxidized concomitantly with its aggregation during its metabolic pathway.

RETRACTED

**Figure 6:** Oxidation of TgMHu2ME199K PrP in Tg mice. PrP^Sc^ in mice, hamsters and human samples cannot be detected by αPrP RVC, demonstrating it is oxidized in it helix3 Met residues. To see if this is also the case for all or part of E200K PrP in the Tg mice, brain homogenates from (wt C57BL/6, TgMHu2ME199K/ko, and scrapie RML), were extracted with sarkosyl and subjected to ultracentrifugation in 10–60% sucrose gradients. Individual fractions of each of the gradients were immunoblotted respectively with α PrP antibodies RTC and RVC. The figure shows that aggregated forms of the mutant protein are not recognized by this antibody, as is the case for RML PrP^Sc^.

### Transmission of spontaneous disease from TgMHu2ME199K to wt mice

Brain samples from heterozygous patients carrying the E200K PrP mutation were shown to transmit prion disease to primates [9] as well as to both wt and TgMHu_2_M PrP mice [10], [28]. To test if our mice also produce infectious prions in addition to fatal spontaneous disease, we inoculated the brain homogenates from an asymptomatic TgMHu2ME199K/wt mouse, from a sick TgMHu2ME199K/wt mouse, as well as from a sick TgMHu2ME199K/ko to groups of wt (C57Bl/6) mice.

We speculated that the presence of a wt allele in the E199K PrP Tgs may induce the formation of some levels of wt PrP^Sc^, thereby facilitating transmission of disease to wt mice following their infection with brains of the Tgs. To this effect, we inoculated the samples from the heterozygous mice only intraperitoneally (i.p.), which although resulting in a longer inoculation time is a less invasive pathway, while the brain homogenate from the sick TgMHu2ME199K/wt was inoculated both i.c. (intracerebrally) and i.p., to maximize the possibility of transmission. As control for the experiment, the brain homogenate of a wt Tg MHu_2_M mouse was inoculated i.p. into a C57B/6 group. These mice were shown previously to remain healthy for more then 640 days [15]. In addition, a wt C57B/6mouse brain homogenate was inoculated i.c. to a group of mice in the same room as a general control for contamination.

RETRACTED

All inoculated animals were evaluated twice a week for clinical signs. Figure 7a shows a typical sick mouse infected with any of the TgMHu2ME199K brain samples, demonstrating lower body atrophy and hind limbs weakness, both properties reminiscence of the spontaneous disease of the donor Tg mice. The transmitted mice also showed “tip toe” walking, a rare feature described only in some prion related models [29]. Clinical signs present in other infectious prion strains, such as kyphosis and plastic tail, were also observed in these mice, as opposed to the donor Tgs. The transmitted disease affected the 6 mice of group 9.9 (inoculated with brain homogenate from a sick TgMHu2ME199K/wt mouse), 3 out of 5 mice of group 9.3 (inoculated with the brain extract from an asymptomatic TgMHu2ME199K/wt mouse), 2 out of the 5 mice inoculated i.c. and 1 out of 6 mice inoculated i.p with a brain extract of a sick TgMHu2ME199K/ko mouse. Disease signs appeared first in the mice infected i.p. with TgMHu2ME199K/wt at about 160–180 days and progressed to their death 2–3 months thereafter (see figure 7c for survival results). After infection with TgMHu2ME199K/ko, some mice became sick at 210 days (i.c) and 300 days (i.p.). While disease in these mice was apparently shorter than in the ones infected with TgMHu2ME199K/wt brains (2–3 weeks), no conclusions can be drown from this observation due to the small numbers. None of the control mice (Tg MHu2M and wt) develop any signs of disease for more than 400 days.

**Figure 7:** Transmission of TgMHu2ME199K prions to wt mice. **a:** Picture of a wt C57BL/6 mouse infected with brain homogenates from TgMHu2ME199K/wt mice showing abnormal hind limb posture. Upper panel shows foot prints of the mice as compared to wt mice, demonstrating abnormal pattern of walking. **b:** Survival curves for wt C57BL/6 mice infected i.p with a TgMHu2ME199K/wt sick mouse brain (group 9.9, close square) or a TgMHu2ME199K/wt asymptomatic mouse brain (group 9.3, open square), as well as i.c (close circles) or i.p (open circles) infected with a TgMHu2ME199K/ko sick mouse brain, or i.p with the brain homogenate of TgMHu_2_M mice (close diamond) and i.c with wt brain homogenate (open triangle). **c:** Brain homogenates of RML infected and wt mice as well as mice (1&2) infected with TgMHu2ME199K/wt brain homogenate (group 9.3) immunoblotted in the presence and absence of PK digestion with α PrP pAb RTC. **d:** Brain homogenates digested in the presence or absence of PK and immunoblotted with α PrP pAb RTC of the brain samples described in table 3. Upper panel: −PK, lower Panel: +PK overdeveloped. Compare sample 1 in figures c and d to appreciate the overdevelopment factor.

RETRACTED

Our results therefore indicate that, like in human E200K brains [10], [28], infectious prions are spontaneously formed in brains of TgMHu2ME199K mice. Most important, potential infectivity is generated in these mice brains before the appearance of clinical signs, as seen by the fact that brains of asymptomatic mice transmitted disease to some of the wt mice. The levels of infectious prions may further increase with disease progression, as seen by the fact that mice infected with the sample from a sick TgMHu2ME199K/wt mice (group 9.9) succumbed to disease in a relative short time, as compared to asymptomatic sample 9.3. Our results also suggest that the wt allele in heterozygous mice may facilitate the transmission of infectivity to naïve wt mice, since transmission from a sick TgMHu2ME199K/ko mice required a very long incubation time and occurred only occasionally, in particular after i.p. inoculation. Facilitation of disease transmission by a wt allele may result from the in-vivo generation of wt PrP^Sc^ in the TgMHu2ME199K/wt mice (even if at marginal levels), concurrently with the quantitative spontaneously generation of mutant disease related PrP. This may indicate that the “species barrier” between both forms of PrP may have been abrogated to some extent in the TgMHu2ME199K/wt mice. It also implies that while wt PrP has little or no effect on the actual presentation of spontaneous disease and its progression, low levels of wt PrP^Sc^ in these animals may be very central for the further passage of disease to naïve wt mice.

### PK resistant PrP in the brains of transmitted wt mice

Figure 7c shows an α PrP immunoblot (pAb RTC) of brain homogenates from individual mice, either infected with scrapie RML, naïve C57B/6, or infected with a brain homogenate from an asymptomatic TgMHu2ME199K/wt mouse, 9.3 (see table 3 for the numbering of samples in figure 7c &d). As can be seen in the figure, sample 1 (derived from sick wt mouse 224 days post infection) presents a similar pattern of disease related PrP as in the RML infected sample, as opposed to, sample 2 (derived from a healthy wt mouse 413 days post infection) in which no PrP^Sc^ can be detected. Figure 7d presents an immunoblots in which individual PK digested samples from infected mice were overdeveloped to allow for the detection of low levels of PK resistant PrP. Consistent with the results in figure 7c, PrP^Sc^ was not be detected in the asymptomatic mice from group 9.3. Contrarily, figure 7d shows that PK resistant PrP forms could be detected in the brains of a selection of brains from mice that succumbed to disease, however the levels and pattern of disease related PrP differed significantly between individual samples (see summary in Table 3). This was true even for extracts of mice infected with the same inoculum, and presenting the same symptoms, as was the case for samples 5–8, which were infected with brain homogenate of a sick TgMHu2ME199K/wt mouse, and samples 9 and 10, both infected with a TgMHu2ME199K/ko brain extract. As opposed to the donor Tg mice, no truncated PrP forms were observed with this antibody in any of the samples. The different levels of PrP^Sc^ in wt mice inoculated with the same prion homogenate are consistent with results from experiments describing the transmission of BSE into wt mice [30]. In that case the presence of PrP^Sc^ in the direct transmission from cow brains could be detected only in about 50% of the mice, while fatal disease presented in all of the animals. PrP^Sc^ became apparent in all mice following adaptation of the new strain by additional mice to mice passages.

RETRACTED

**Table 3:** Summary of transmission studies.

sample	group	PK resistant PrP	Age of death (days)
1	Infected with Tg/wt 9.3 (i.p)	+++	224
2	Infected with Tg/wt 9.3 (i.p)	−	Sac at 413
3	Infected with Tg/wt 9.3 (i.p)	−	Sac at 413
4	Infected with Tg/wt 9.3 (i.p)	−	Sac at 413
5	Infected with Tg/wt 9.9 (i.p)	+++	224
6	Infected with Tg/wt 9.9 (i.p)	+++	252
7	Infected with Tg/wt 9.9 (i.p)	+	254
8	Infected with Tg/wt 9.9 (i.p)	+	257
9	Infected with Tg/KO (i.c)	+++	210
10	Infected with Tg/KO (i.c)	+/−	210
11	TgMHu2ME199K/KO	++	Sac at 240
12	TgMHu2ME199K/wt	++	Sac at 240
13	wt C57Bl/6	−	Sac at 240
14	Mouse RML	+++	180

This table summarizes the results of the transmission experiment as described in figure 7 b (survival of mice), as well as the presence of PK resistant PrP in infected samples (panels c &d).

### Neuropathological evaluation of wt mice infected with TgMHu2ME199K brains

Sections of formalin-fixed, paraffin-embedded brains of mice infected with TgMHu2ME199K/wt, TgMHu2ME199K/ko and RML prions were examined for prion parameters. Figure 8a presents sections of the frontal cortex. Brains infected with TgMHu2ME199K samples present minor to moderate spongiform changes, distinctly different from the high levels of spongiform changes apparent in the RML strain [31]. The infected mice also showed severe astrogliosis and neuronal loss, as well as prominent diffuse synaptic type disease-related 6H4 PrP immunoreactivity, similar to the ones seen for the RML sections. As opposed to the spontaneous disease of TgMHu2ME199K mice (figure 3), only low levels of RTC related immunostaining were observed in the infected mice's brains, as shown in figure 8a for the sample infected with a TgMHu2ME199K brains. RTC immunostaining was not observed in the RML samples.

RETRACTED

**Figure 8:** Transmission of TgMHu2ME199K prions to wt mice: pathology. **a:** Frontal cortex sections of mice infected with RML or with TgMHu2ME199K prions on a wt or ablated background, analyzed for prion pathological properties, spongiosis, gliosis, and disease related PrP immunoreactivity with pAb RTC and mAb 6H4. Scale bar in upper left image indicates 50 µm. **b:** RTC immunoreactivity in the absence of formic acid for brains infected with TgMHu2ME199K/wt or RML, as well as for naïve PrP ablated mice. Picture shows different pattern of immunoreactivity for both infected samples. Scale bar in upper left image indicates 20 µm.

To test whether RTC related immunostaining can distinguish better between the RML and TgMHu2ME199K generated prions at a different experimental setup, we immunostained sections of TgMHu2ME199K and RML infected mice with RTC following a less harsh epitope revealing treatment (no formic acid after heating with citrate). Figure 8b shows that under these conditions, pAb RTC detected intracellular PrP aggregates in the mice infected with TgMHu2ME199K, but not in those infected with RML homogenates. Both brain samples presented a diffused immunoreactivity reminiscence of PrP^C^. No immunoreactivity of any kind was observed in brains of PrP ablated mice, indicating that the positive stain in the infected sample is indeed PrP.

In conclusion, clinical, biochemical and pathological results presented in this section demonstrate that brains from TgMHu2ME199K mice may generate de-novo prions with specific properties. These prions may readily transmit to wt mice, and are particularly infectious when in the brains of sick TgMHu2ME199K on a wt background. Whether other organs of these mice, and in particular blood and immune cells, may also transmit infectivity remains to be established. Results from such experiments may be very important to assess blood safety in the community.

## Discussion

Constructing a clinically relevant mouse model has proven to be a hard task for most neurodegenerative diseases [32]. The existing models, in particular for Alzheimer's of Parkinson diseases present mostly pathological markers and in some cases behavioral changes, but not obvious clinical symptoms, or age dependent deterioration that correlates with those observed in human patients [33].

As opposed to models for the more common neurodegenerative conditions, several genetic prion diseases linked to pathological mutations in the *PRNP* gene have been reconstructed clinically in transgenic mice lines. Each of these models demonstrate several of the basic features of genetic fatal prion disease, as is the case for those mimicking GSS linked to the PrP P101L mutation [3] [21], the D177N CJD or FFI mutations [18], [19] or the insertional PrP modification [34]. These mouse models were seminal in proving that spontaneous prion disease may indeed result from the presence of a pathological PrP mutation.

RETRACTED

In this work, we describe the properties of a Tg line mimicking the most common genetic prion disease [3], i.e CJD linked to the human E200K PrP mutation. Our Tg line presents all prion relevant properties, spontaneous fatal disease, PrP pathology and transmission of prion disease to wt mice. This is particularly intriguing in view of the fact that two other models of this same mutation failed to generate disease in transgenic mice. While they may be other explanations for the different results in our case, we assume that the introduction of the E200K mutation into a chimeric mouse human PrP, as opposed to a mouse PrP [21] or a human PrP [20], is of biological importance. Chimeric PrP may constitute the bridge that allows human prion diseases to manifest in mice. Indeed, chimeric human mouse PrP was required to transmit at low incubation times genetic and sporadic human prion disease to mice [15]. Moreover, while Tgs expressing the GSS 102 mutation in human PrP did not present spontaneous disease, the same mutation in chimeric PrP did present neurodegenerative disease [28]. Whether the structure of chimeric PrP is more favorable for disease transmission or otherwise the chimeric form has the ability to bind a mouse component important for transmission of human prion diseases to mouse models remains to be established.

Another novel feature of our Tg line is the generation of de-novo infectious prions that could be transmitted to naïve wt mice. Indeed, E200K CJD is the genetic disease most similar to the sporadic forms, in both clinical appearance, age of onset and pathology [2], [10]. This may imply that E200K de-novo prions are more similar in structure to sporadic ones, which are highly transmissible [9]. Whether the chimeric background of E200K PrP in these mice is also a factor in the transmissibility of disease is unknown at this point, however it is important to state that chimeric mouse human PrP Tg mice are susceptible for infection with both mouse and human prions [28].

While the neuropathology features of our Tg mice were similar to E200K human patients with regard to reduced spongiosis and intracellular PrP accumulation [24], PK resistant PrP in the TgMHu2ME199K mice was detected mostly by the C-terminal pAb RTC, suggesting a considerable fraction of disease related PrP in the brains of these mice accumulates as a truncated form. Indeed, diverse truncated PrP forms were also described in brains of CJD patients [35], including those carrying the E200K mutation [36]. Interestingly, intraneuronal immunoreactivity in these CJD patients predominates in the brainstem and may be associated with alterations in the accumulation of other neurodegeneration-related proteins (e.g. phospho-tau, alpha-synuclein) [24]. Evaluation of concomitant protein pathology in our model is the objective of another ongoing study.

RETRACTED

Because gCJD is a dominant genetic disorder, we investigated the properties of the TgMHu2ME199K mice not only on a PrP ablated but also on a wt PrP background. We first speculated that the presence of wt PrP may preclude some disease symptoms related to the absence of the elusive PrP^C^ activity or to the putative toxicity of truncated PrP forms, as was shown previously in other systems [29]. However, this is probably not the case, as can be inferred from the fact that no significant differences were seen between both lines of Tg mice in clinical symptoms, kinetics and pathological examination. Finally, while the investigation of a small group of homozygous E200K CJD patients showed a moderate decrease in the age of disease onset for most patients, it also described a patient with a very slow progressive disease (96 months), who died in the absence of PrP^Sc^ accumulation [37]. Whether disease onset in one or both lines of TgMHu2ME199K mice may be modulated by oxidative stress or other pathogenic insults is under investigation in our laboratory.

In summary, we believe that our TgMHu2ME199K lines will play a central role both in the elucidation of genetic prion disease pathogenic mechanism as well as in the search for anti-prion compounds. The early presence of spontaneous disease followed by their sequential age related deterioration during several months until death will permit to study the long term effect of reagents that may delay disease onset in at risk subjects. Among those to be tested first are substances suggested to have a marginal but still encouraging result in already sick CJD patients, such as doxicyline [38] and flupirtine [7], as well as those believed to present significant therapeutic results in scrapie infected mice or infected cells, such as Quinacrine and Simvastatin [39], [40]. Novel approaches such as passive [41] or active immunization, as well as RNAi inhibition of mutant PrP expression [42], will also be tested in the near future.

## Materials and Methods

### Ethical statement

This study was carried out in strict accordance with the recommendations in the Guide for the Care and Use of Laboratory Animals of the National Institutes of Health. The protocol was approved by the Committee on the Ethics of Animal Experiments of the Hebrew University Medical school (Permit Number: MD-11746-5). All surgery was performed under sodium pentobarbital anesthesia, and all efforts were made to minimize suffering.

RETRACTED

### Generation of TgMHu2ME199K mice

Transgenic mice harboring the E200K mutation were generated by one of us (ZM) in the Prusiner laboratory as follows. Using site-directed mutagenesis by PCR, the E200K mutation was inserted into the chimeric human/mouse PrP open reading frame (ORF) of an MHu_2_M construct that was previously prepared as described [15]. The 0.8 kb SalI-XhoI fragment containing the PrP ORF with the E200K mutation was inserted into cos.ShaTet and further injected into transgenic mice ablated for the PrP gene [43]. Creating and screening of the transgenic mice were done as described [44]. Several lines were produces at the time and at least 2 presented spontaneous prion disease (ZM, personal communication). For the present project, C57BL/6 female mice were impregnated with frozen sperm from one of these lines in the Jackson laboratories. The designated offspring were subsequently crossed either with wt or with PrP ablated C57BL/6 mice (Harlan laboratories, obtained by crossing of PrP^0/0^ FVB mice [43] with the C57BL/6 strain for 10 generations, and screened for the presence of the TgMHu2ME199K PrP, ablated or wt PrP allele, as required. The mice used in this project are of a mixed C57B/6/FVB background, ranging from 75- to 95% C57B/6.

### Real time PCR

Total RNA from mice brains was isolated using TRI reagent (Sigma, Israel). cDNA was prepared from 2 µg of total RNA using MuLV reverse transcriptase and random hexamers (Promega) according to the manufacturer's instructions. Quantitative RT-PCR was carried out in 15 µl reactions containing 1 µl of cDNA, 0.3 µM of the appropriate primers (sigma, Israel), and 7.5 µl of the SYBR Green master mix (Finnzymes). Gene amplification was carried out using the GeneAmp 7500 Sequence Detection System (Applied Biosystems). Measurements were performed in triplicates and UBC (Ubiquitin C) and TBP (TATA-box binding protein) transcript levels were used to normalize between samples. The primers used were PrP, 5′-CAA GCA GCA CAC GGT CAC C-3′ (forward), 5′-GGC CTG GGA CTC CTT CTG G-3′ (reverse) **TBP**, 5′-TGT GCA CAG GAG CCA AGA-3′ (forward), 5′-CCC CAC CAT GTT CTG GAT-3′ (reverse); UBC, 5′-CAG CCG TAT ATC TTC CCA GAC T-3′ (forward); 5′-CTC AGA GGG ATG CCA GTA ATC TA-3′ (reverse). The primers used for PrP were chosen so that they can be used for both wt (mouse) PrP as well as for MHu_2_M PrP.

RETRACTED

### Spontaneous disease in the TgMHu2ME199K mice

Mutant TgMHu2ME199K mice from both lines (PrP ablated or wt background) were followed twice a week for the appearance of spontaneous neurological disease. Mice were scored for disease severity and progression according to the scale of clinical signs described in Table 2. This scale was designed by us to fit the clinical symptoms observed in the Tg mice and was proven to be parallel to the NNS (neurological severity score). Mice were sacrificed according to the ethical requirements of the Hebrew University Animal authorities (when too sick or paralyzed to reach food and water, or after loosing 20% body weight).

### Clinical and behavioral evaluation

As described in table 2 mice were scored for disease severity and progression according to a scale of clinical signs designed by us to fit the clinical symptoms observed in the Tg mice. Hind limbs weakness was first evaluated by closely watching the mouse walking on a flat surface looking for sings of abnormal limb posture or abnormal walking pattern (high or low gait, leg dragging). Next, mice were tested for their ability to walk on a 3 cm beam in a straight line and maintain balance. Finally mice were lifted by their tail to check for leg clasping. Full paralysis was evaluated by total lack of movement in the limb. This scale of scoring was proven to be parallel to the NSS (neurological severity score) [45]. Blindness was tested by the lack of reaction of the mice to a paper slowly placed before its eyes.

### Transmission of disease from TgMHu2ME199K mice to wt mice

10% brain homogenates of asymptomatic or sick TgMHu2ME199K/wt, sick TgMHu2ME199K/ko, as well as from control TgMHu_2_M and naïve wt mice were each inoculated i.p. or i.c, as designated in the text, into a group of 6 C57BL/6 mice (Harlan laboratories). The inoculated mice were scored twice a week for clinical signs of prion disease until the beginning of symptoms and more closely thereafter. Following termination of each experiment, mice were sacrificed and analyzed for pathology and for the presence of disease related PrP.

### Pathology

Four µm thick sections of formalin fixed, paraffin embedded brains of TgMHu2ME199K mice as well as of C57BL/6 mice infected with TgMHu2ME199K brains, in addition to controls and PrP ablated mice were evaluated for the presence of disease related PrP, gliosis and spongiform changes as previously described [24]. A less harsh epitope retrieval method, with the avoidance of formic acid, was also applied in some cases.

### Immunoblotting of brain homogenates from TgMHu2ME199K mice

Brains from TgMHu2ME199K mice on a wt or ablated background, normal mice, control TgMHu_2_M and scrapie RML infected mice were homogenate at 10% (W/V) in 10 mM Tris-HCl, pH 7.4 and 0.3 M sucrose. For Proteinase K digestions, 30 µl of 10% brain homogenates extracted with 2% sarkosyl were incubated with 30 µg/ml Proteinase K for 30 min at 37°C. Samples were subsequently subjected to SDS PAGE and immunoblotted with the diverse α-PrP antibodies, as described in Figure 2 a. Protein precipitation experiments, as the ones observed in Figure 5 c, were performed by ultracentrifugation of Sarkosyl extracted homogenates at 100000 g, and subsequently separating pellets from supernatant. Deglycosylation by PNGase was performed as previously described [46].

RETRACTED

### Sucrose gradient centrifugation experiments

Normal and prion infected Sarkosyl extracted brain homogenates were subjected to sucrose gradients as described [47]. Shortly, 140 µl of 10% brain homogenates extracted in the presence of 2% Sarkosyl were overlaid on a sucrose gradient composed of layers of increasing concentrations of sucrose (10–60%). Gradients were then centrifuged for 1 h at 55000 rpm in a Sorval mini-ultracentrifuge and subsequently 11 samples of 120 µl were collected from the top to the bottom. Gradient fractions were then immunoblotted with either α PrP pAb RTC or RVC.

### Accession numbers

1. prnp mus musculus: ENSMUST00000091288
2. prnp homo sapiens: ENSG00000171867
3. UBC mus musculus: ENSMUSG00000008348
4. TBP mus musculus: ENSMUSG00000014767

## Supporting Information

Figure S1 **Time course histopathology and PrP immunoreactivity in the brain and spinal cord of TgMHu2ME199K mice.** **a:** Hematoxylin & Eosin (H&E) staining of frontal cortex: Spongiform change was noted only focally in end-stage animals (H&E staining, frontal cortex). **b–d:** GFAP staining: Reactive astrogliosis progressed with the age of the animals as represented here in the frontal cortex (**b**), thalamus (**c**), and the spinal cord (**d**). **e** & **f:** PrP immunoreactivity. PrP immunoreactivity at disease end point is presented with 2 α PrP antibodies, pAb RTC and mAb 6H4, in different brain areas. For comparison the right lower image is a representative micrograph of intraneuronal PrP immunoreactivity in the putamen in human genetic CJD associated with E200K mutation using αPrP mAb 12F10. Bar in upper left image represents 50 µm for all upper panel images and 20 µm for lower panel images.
(TIF)
